The article "The effect of marathon on mRNA expression of anti-apoptotic and pro-apoptotic proteins and sirtuins family in male recreational long-distance runners" was retracted in 2014. Reason: errors in the images.

# The effect of marathon on mRNA expression of anti-apoptotic and pro-apoptotic proteins and sirtuins family in male recreational long-distance runners

**DOI:** 10.1186/1472-6793-10-7

**Published:** 2010-05-12

**Authors:** Gabriella Marfe, Marco Tafani, Bruna Pucci, Carla Di Stefano, Manuela Indelicato, Angela Andreoli, Matteo Antonio Russo, Paola Sinibaldi-Salimei, Vincenzo Manzi

**Affiliations:** 1 Department of Experimental Medicine and Biochemical Sciences, University of Rome "Tor Vergata" Via Montpellier 1, 00133, Rome, Italy; 2 Department of Cellular and Molecular Pathology, IRCCS San Raffaele Pisana, Via dei Bonacolsi snc, 00163, Rome, Italy; 3 Human Nutrition Unit, University of Rome "Tor Vergata" Via Montpellier 1, 00133, Rome, Italy; 4 Department of Experimental Medicine, La Sapienza University, Viale Regina Elena 324, 00161, Rome, Italy; 5 School of Sport and Exercise Sciences, University of Rome Tor Vergata" Via Columbia s.n.c. 00133 Rome, Italy

## Abstract

**Background:**

A large body of evidence shows that a single bout of strenuous exercise induces oxidative stress in circulating human lymphocytes leading to lipid peroxidation, DNA damage, mitochondrial perturbations, and protein oxidation.

In our research, we investigated the effect of physical load on the extent of apoptosis in primary cells derived from blood samples of sixteen healthy amateur runners after marathon (a.m.).

**Results:**

Blood samples were collected from ten healthy amateur runners peripheral blood mononuclear cells (PBMCs) were isolated from whole blood and bcl-2, bax, heat shock protein (HSP)70, Cu-Zn superoxide dismutase (SOD), Mn-SOD, inducible nitric oxide synthase (i-NOS), SIRT1, SIRT3 and SIRT4 (Sirtuins) RNA levels were determined by Northern Blot analysis. Strenuous physical load significantly increased HSP70, HSP32, Mn-SOD, Cu-Zn SOD, iNOS, GADD45, bcl-2, forkhead box O (FOXO3A) and SIRT1 expression after the marathon, while decreasing bax, SIRT3 and SIRT4 expression (P < 0.0001).

**Conclusion:**

These data suggest that the physiological load imposed in amateur runners during marathon attenuates the extent of apoptosis and may interfere with sirtuin expression.

## Background

Apoptosis, or programmed cell death, is a normal physiological function essential for the homeostasis of immuno haemopoietic tissues. This process occurs via specific signaling pathways, eventually leading to DNA fragmentation, nuclear condensation, proteolysis and cell fragmentation [1]. An important regulatory event in the apoptotic process is the activation of caspases, a family of cysteine proteases, which regulate two major and relatively distinct pathways, the extrinsic and intrinsic pathways. The extrinsic pathway known also as mitochondrial pathway involves pro- and anti-apoptotic members of the bcl-2 family of proteins [2,3].

The initiation of apoptosis is dependent on a variety of signals, many of which can be modulated by strenuous exercise [4-7]. Consequently, it has been suggested that apoptosis contributes to the loss of blood lymphocytes after exercise possibly via the cell surface death receptor CD95 (Fas/Apo-1) signaling [8-10], resulting in post-exercise lymphocytopenia, which could lead to lowered immunity in athletes performing frequent and physically demanding training regimens. Studies that have examined the effects of exercise on the extent of apoptosis in blood lymphocyte in humans are few, thus making it difficult to draw any definitive conclusions [8-12].

Exercise increases oxygen consumption and causes a disturbance of intracellular pro-oxidant-antioxidant homeostasis [13]. The mitochondrial electron transport chain [14], and xanthine oxidase [15] have been identified as major sources of intracellular reactive oxygen species (ROS) and free radical generation during exercise [15]. Two recent studies have proven that ROS accumulation readily modifies the activity of a new class of proteins called sirtuins [16,17].

In humans the sirtuins family of proteins is composed of seven members (SIRT1 through 7) that share the catalytic domain with Sir2 [18,19]. In particular, SIRT1 can modulate cellular stress response and survival through regulation of p53 [20-22], NF-kB signaling [23] and FOXO transcription factors [24,25]. Several studies showed that SIRT1 is a key regulator of cellular metabolism [26] and survival in response to external stressors [27]. Furthermore, since skeletal muscle increased levels of oxidative damage with aging [28,29], regular exercise is very useful in increase its antioxidant potential that can be modulated by the activity of SIRT1 [28-31]. Recent studies have reported that others sirtuins, such as SIRT3, SIRT4 and SIRT5, are located in the mitochondria [32,33]. In particular, it has been demonstrated that the mitochondrial NAD-dependent deacetylase SIRT3 plays a role in the maintenance of basal ATP levels and as regulator of mitochondrial electron transport [34]. In fact, SIRT3 decreases mitochondrial membrane potential and reactive oxygen species production, while increasing cellular respiration [35].

The present investigation has been designed to test the effect of an endurance effort, typical in runners participating in standard (42 km) marathon events, on apoptotic cell status in a controlled laboratory setting. Furthermore, we have studied the effect of the same endurance effort on sirtuin proteins in order to understand their role in this kind of exercise.

## Results

### Marathon race

All subjects successfully completed a marathon (n = 10). Total TRaining IMPulse (TRIMP) score accumulated over the marathon race averaged 523 ± 67 arbitrary unit, equivalent to exercise at 80% of heart rate reserve for 200 to ~220 min.

### Exercise and bcl-2 pathway apoptotic signaling

We determined the effects of exercise on bcl-2 family upstream of caspase-3, including caspase-9 and bax: bcl-2 ratio. Figure 1 shows the same procaspase-9 RNA levels in the group before and after marathon (b.m. and a.m.). RNA expression of proapoptotic bax in the group showed a significant decrease after marathon (Figure 2B). By contrast, the antiapoptotic bcl-2 RNA levels increased in the group after marathon (Figure 2B) (Table 1). Thus, we calculated bax: bcl-2 ratio in the same group before and after marathon and such ratio was attenuated after marathon (Figure 2B, C).

**Figure 1:** **Effects of marathon on procaspase-9 mRNA expression**. Procaspase-9 mRNA content was estimated by Northern Blot. **(A) **RNA was extracted, electrophoresed and hybridized with a labelled probe as described under Methods. β-actin was used as loading control. Blot is representative of three separate experiments. (P < 0.0001)

**Figure 2:** **Effects of marathon on bax and bcl-2 mRNA expression**. A) bax and bcl-2 RNA content was estimated by Northern Blot. RNA was extracted, electrophoresed and hybridized with a labelled probe for bax and bcl-2 as described under Methods. β-actin was used as loading control. Blots are representative of at least three separate experiments. (P < 0.0001). B) bax: bcl-2 ratio in samples before marathon and after marathon was obtained by densitometry analysis of the blots shown in A. C) Change bax: bcl-2 ratio in samples before and after marathon.

**Table 1:** Changes of different genes expression before marathon and after marathon.


	**Before marathon**	**After marathon**	**Mean difference**	**95% CI Lower - Upper**	**Magnitude of the difference**	
				
	**Mean ± SD**	**Mean ± SD**			**Effect size**	**Interpretation**

bax	3.35 ± 0.91	0.60 ± 0.21	-2.75*	-3.43 to -2.07	0.90	large
bcl-2	0.91 ± 0.21	3.25 ± 1.17	2.34*	1.56 to 3.12	0.83	large
Cu-Zn SOD	0.69 ± 0.25	3.50 ± 0.74	2.81*	2.25 to 3.37	0.93	large
HSP70	1.27 ± 0.53	3.65 ± 1.31	2.38*	1.73 to 3.02	0.88	large
iNOS	0.95 ± 0.08	4.10 ± 0.66	3.15*	2.67 to 3.63	0.96	large
Mn-SOD	0.52 ± 0.30	5.20 ± 1.11	4.68*	3.73 to 5.63	0.93	large
SIRT1	1.12 ± 0.28	3.60 ± 0.69	2.48*	1.90 to 3.06	0.91	large
SIRT3	0.97 ± 0.26	0.18 ± 0.11	-0.79*	-0.98 to -0.59	0.90	large
SIRT4	1.11 ± 0.25	0.20 ± 0.13	-0.91*	-1.14 to -0.68	0.90	large
Ratio bax: bcl-2	2.10 ± 0.19	0.87 ± 0.27	-1.23*	-1.43 to -1.03	0.96	large

* = Significant difference between before and after marathon (P < 0.0001); 95% CI = 95% confidence intervals of the difference

### DNA laddering

Representative DNA fragmentation is shown in Figure 3. A laddering pattern was observed in DNA isolated from samples in which the ratio bax: bcl-2 after marathon was slightly higher than the others. By contrast, we did not observe any apparent laddering pattern in the DNA isolated from those samples in which the ratio bax: bcl-2 was lower than the others.

**Figure 3:** **DNA laddering**. Samples 2, 3, 6, 7 and 10 from Figure 2 were collected before and after marathon and processed for DNA fragmentation as described under Methods.

### HSP70, HSP32, Cu-Zn-SOD, and Mn-SOD, i-NOS levels

Northern blot analysis demonstrated that the RNA content of HSP70, HSP32 increased substantially in the studied group after marathon (Figure 4). Similarly, the RNA content of Cu-Zn-SOD, Mn-SOD and i-NOS increased after marathon (Figure 4). We have found that the change in HSP70 RNA expression is positively correlated to the change of both Mn-SOD (r = 0.93; P = 0.001; 95% CI: 0.98 to 0.73; ES 0.71) and bcl-2 transcripts (r = 0.84; P = 0.002; 95% CI: 0.96 to 0.45; ES 0.2) after marathon (Fig. 5). In addition, we have also found that the change in HSP32 RNA expression is positively correlated to the change of bcl-2 transcripts (r = 0.82; P = 0.003; 95% CI: 0.96 to 0.41; ES 0.2) (Figure 5).

**Figure 4:** **Effects of marathon on the Cu-Zn-SOD, Mn-SOD, i-NOS, HSP70 and HSP32 mRNA expression**. Cu-Zn-SOD, Mn-SOD, i-NOS, HSP70 and HSP32 RNA levels were estimated by Northern Blot. RNA was extracted, electrophoresed and hybridized with a labelled probe as described under Methods β-actin was used as loading control. Blots are representative of at least three separate experiments (P < 0.0001)

**Figure 5:** **Relationships between change in HSP70, HSP32, Mn-SOD and bcl-2 RNA expression after marathon**. The HSP70 content is positively correlated to both Mn-SOD and bcl-2 transcript contents after marathon. (P < 0.0001)

### SIRT1, SIRT3 and SIRT4 levels

Northern blot analysis demonstrated that the RNA contents of SIRT1 increased substantially in the group after marathon (Figure 6). On the other hand, the RNA contents of SIRT3 and SIRT4 decreased in the group after marathon (Figure 6). Furthermore, we also found a significant positive correlation between a change in SIRT3 RNA levels and TRIMP (r = 0.76; P = 0.03; 95% CI: 0.94 to 0.11; ES 0.99) after marathon (Table 2). A trend of correlation was detected between the TRIMP and change in SIRT4 RNA levels after marathon (r = 0.68, P = 0.06).

**Table 2:** Pearson correlation (*r*) between TRIMP, SIRT3 and GADD45

		**SIRT3**			**GADD45**	
		
	**r**	**CI (95%) Upper - Lower**	**Effect size**	**r**	**CI (95%) Upper - Lower**	**Effect size**
		
TRIMP	0.76*	(0.94 to 0.11)	0.99	0.79**	(0.95 to 0.32)	0.99

*Abbreviations*: TRIMP, Training Impulse; *P < 0.03; **P < 0.006

**Figure 6:** **Effects of marathon on SIRT1, SIRT3 and SIRT4 in mRNA expression**. SIRT1, SIRT3 and SIRT4 RNA levels were estimated by Northern Blot. RNA was extracted, electrophoresed and hybridized with a labelled probe as described under Methods β-actin was used as loading control. Blots are representative of at least three separate experiments. (P < 0.0001)

In addition, Northern blot analysis showed that RNA levels of the SIRT1-dependent transcription factor FOXO3A and its target GADD45 were increased in the studied group after marathon (Figure 7). In addition, we found also a significant positive correlation between a change in GADD45 RNA levels and TRIMP (r = 0.79; P = 0.006; 95% CI: 0.94 to 0.32; ES 0.98) after marathon (Table 2).

**Figure 7:** **Effects of marathon on the GADD45 and FOXO3A in mRNA expression**. GADD45 and FOXO3A RNA levels were estimated by Northern Blot. RNA was extracted, electrophoresed and hybridized with a labelled probe as described under Methods β-actin was used as loading control. Blots are representative of at least three separate experiments. (P < 0.0001)

## Discussion

The present study provides evidence that strenuous physical load attenuates the extent of apoptosis in amateur runners. In particular, we found that both HSP70 and HSP32 RNA expression is positively correlated to bcl-2 transcript content after marathon (Figure 5). We can suppose that HSP70 and HSP32 may play an anti-apoptotic role in modulating the homeostasis of apoptotic factors in amateur runners after exercise. A critical step in the execution of the apoptotic program is cleavage of caspases [36]. The RNA levels of procaspase-9 were not changed in the amateur runners before and after marathon. Combined with DNA fragmentation data, this is the first direct evidence that strenuous physical load endured during marathon provides a physiological protection against the proapoptotic process.

It has also been suggested that ROS production influences apoptosis mainly through the modulation of the mitochondrial mediated pathway [37]. It has been hypothesized that a high oxidative stress level destabilizes the mitochondrial membrane homeostasis and therefore induces the formation of mitochondrial membrane permeability pores releasing pro-apoptotic factors (e.g., cytochrome *c*). Bcl-2 family proteins are known to be responsible for the modulation of mitochondrial membrane pore formation and therefore regulating mitochondrial-mediated apoptosis. We have shown that RNA levels of proapoptotic bax were consistently decreased after marathon, whereas, RNA levels of antiapoptotic bcl-2 were slightly increased after marathon thereby causing a decreased bax: bcl-2 ratio (Figure 2B, C). Our findings are consistent with the hypothesis that alterations in bax: bcl-2 ratio with exercise regulate downstream caspase-driven apoptosis during the exercise. Furthermore, Ferrer and colleagues (2009) [38] reported a decreased expression of bcl-2 after intense exercise versus the expression obtained previous exercise. The differences with our data could be attributed to differences between both experiments as the type of exercise, duration of the tests, time after exercise of sampling, differences between the moment in which the sampling was made before exercise. We have examined the possibility that the age range and the differences in VO_2 _max of our subjects could influence the apoptotic parameters considered. However, we did not find any significant correlation between differences in age or VO_2 _max and all the molecular parameters measured (data not shown).

Several antioxidant enzymes, including Cu-Zn-SOD, catalase, glutathione peroxidase, glutathione reductase, and mitochondrial Mn-SOD have been implicated as crucial endogenous antioxidant enzymes in biological systems. In the present study, we have demonstrated that the RNA content of Mn-SOD increases after marathon (Figure 4). These observations suggest that the answer of the cell may attenuate apoptosis. Our data are consistent with the idea that an increased antioxidant capacity and modulated oxidative stress from strenuous physical load may be involved in reducing pro-apoptotic genes.

HSPs are a group of highly conserved proteins induced by a variety of stresses, including hyperthermia, pH disturbance, and oxidative stress. There is evidence supporting the hypothesis that HSP70 inhibits apoptosis by modulating the mitochondrial-mediated pathway [39-41]. Li and colleagues (2000) [40] reported that HSP70 inhibits apoptosis by suppressing the formation of apoptosomes due to an effect downstream of cytochrome *c *release and upstream of caspase-3 activation. Beere and colleagues (2000) [39] have shown that HSP70 inhibits apoptosis by preventing the recruitment of procaspase-9 to the apoptosome. Furthermore, Fehrenbach et al. (2003) [42,43] have shown that the protective functions of HSPs include antioxidative and antiapoptotic effects and may prevent damage to DNA. Here, we have found a significant relationship between HSP70 and bcl-2 RNA (Figure 5) levels following marathon, but the underlying cellular and molecular mechanisms involved in this exercise induced adaptations in apoptosis and HSP70 are unknown and require further investigation.

Furthermore, in the present study we demonstrate, for the first time, that SIRT1 mRNA expression increases after marathon (Figure 6). It is therefore very likely that increased SIRT1 expression by endurance exercise results in elevated SIRT1 deacetylase activity as well as causing an allosteric effect of an increased cytosolic NAD^+^-to-NADH ratio.

In addition, an increase in SIRT1 mRNA levels could exert an antioxidant effect. Brunet et al. [34] demonstrated that in mammalian cells SIRT1 appears to control the cellular response to stress by regulating FOXO transcription factors that function as sensors of the insulin signaling pathway and as regulators of longevity. In particular, these authors showed that SIRT1 and FOXO3A form a complex in response to oxidative stress stimulus [24]. Mammalian FOXO factors control several biological functions, such as cell cycle arrest, detoxification of ROS [44] and repair of damaged DNA [45]. SIRT1 increased FOXO3A ability to induce cell cycle arrest and enhanced expression of a FOXO3A target involved in DNA repair, such as GADD45 [24]. Because it is known that exercise training exerts its beneficial effects particularly on the cardiovascular system, we tested FOXO3A and its targets involvement in group, showing that exercise training enhanced FOXO3A RNA levels. This was associated with an increase in GADD45 mRNAs after marathon. This finding could be related to higher oxidative stress in samples that would induce to choose apoptosis or necrosis rather than repair as mechanism of detoxification.

Furthermore, we found that SIRT3 and SIRT4 RNA levels decreased after marathon and also that there was a positive correlation between SIRT3 RNA levels and training load (Table 2) [38]. A trend of correlation was also detected between the TRIMP and change in SIRT4 RNA levels after marathon, however this trend was not statistically significant (P = 0.06). These two sirtuin proteins are known to localize in the mitochondria; although SIRT3 was reported to change its localization from mitochondrial to nuclear when coexpressed with SIRT5 [46,47]. The recent identification of the first substrates for mitochondrial sirtuins--acetyl coenzyme A synthetase 2 [48,49], and glutamate dehydrogenase (GDH) [32]--as targets of sirtuins 3 and 4, respectively, revealed that these sirtuins control a regulatory network that has implications for energy metabolism and the mechanisms of caloric restriction (CR) and lifespan determination [20]. In particular, SIRT3 has a role for the mitochondrial NAD-dependent deacetylase, for the maintenance of basal ATP levels and as a regulator of mitochondrial electron transport [34]. Considering our preliminary results and the fact that little is known about the role of SIRT3 and SIRT4 in human physiology, the differences in SIRT3 and SIRT4 mRNA expression before and after marathon that we observed may be due to the redox changes in the mitochondria during the marathon stress. Thus, our results support the hypothesis that exercise may interfere with expression of this family of proteins at mitochondrial level. Further studies are under way to study this aspect.

## Conclusion

Our data presented in this study show that: 1) the balance between pro and anti-apoptotic genes is shifted to a anti apoptotic state after strenuous exercise 2) strenuous exercise may interfere with expression of SIRT3 and SIRT4, which may be a key regulator of exercise training. Additional studies are under way in order to elucidate the role of the SIRTs family and bcl-2 family during different exercise protocols.

## Methods

### Study design and ethical approval

Subjects underwent a baseline testing session in an exercise laboratory. Seven days prior to the treadmill runs which were conducted at a local private gymnasium. The study was cleared by the Institute's Ethics committee and informed written consent was obtained from all the participants.

The study protocol conformed to the guidelines of the Helsinki Conference for research on human subjects.

### Subject characteristics

Sixteen healthy, well-trained, male recreational long-distance runners were selected from volunteers who offered to take part in this study (additional file 1). The mean physiological and anthropometric characteristics of the ten male subjects are shown in Table 3. Selection criteria included an age range between 30 and 53 years, the absence of clinical signs or symptoms of infection, cardiovascular disease or metabolic disorders and a minimum weekly training distance. Subjects were also asked to refrain from ingesting additional nutrient supplements, analgesics, anti-inflammatory drugs, caffeine or alcohol for at least 24 h prior to the trial run. Six subjects, which did not participate in the marathon, were considered control for transcripts of the genes examined and DNA fragmentation (additional file 1, 2, and 3).

**Table 3:** Body composition and physiological parameters of the subjects


**Variables**	**Mean ± SD**

Age (years)	42.00 ± 7.38
Height (m)	1.78 ± 0.06
Body mass (Kg)	74.54 ± 7.70
Fat free mass (Kg)	64.04 ± 4.71
Fat mass (Kg)	10.50 ± 5.68
BMI (Kg/m^2^)	23.58 ± 2.48
Total body water	46.86 ± 3.43
HR_max _(beat·min^-1^)	183.80 ± 3.82
HR_rest _(beat·min^-1^)	51.00 ± 3.40
VO_2max _(ml·kg^-1^·min^-1^)	60.17 ± 3.25

Information on prior race experience, dietary preparation and expected finishing time was obtained with a self-administered questionnaire before the race. The amateur runners were requested to maintain a standardised diet for one month before the marathon and were given an activity diary. The macronutrient composition of the meal provided carbohydrate (65%), protein (15%) and fat (20%). Food and fluid intake during the race was evaluated by direct observation by trained research assistants.

### Body composition analysis

Body composition, fat-free mass (FFM), fat mass (FM), total body water (TBW) were assessed using bioelectrical impedance analysis (BIA). BIA measurements were performed in the morning after an overnight fast of at least 12 h, abstinence of alcohol consumption for 48 h and absence of strenuous physical activity for 24 h before the testing day. Participants emptied their bladders within 30 min before undergoing the measurements. All measurements were performed on the dominant side, while participants lied supine on an examination table with their limbs abducted away from the trunk. Four gel electrodes were attached on defined anatomical positions on the hand, wrist, ankle and foot [50,51]. The BIA measurements were performed using an Akern BIA (Florence, Italy) and Littmann 2325VP adhesive electrodes (3M, St Paul, MN, USA).

### Fitness assessment and quantification of marathon physical load

In the week before the marathon, maximal oxygen uptake (VO_2max_) was determined using an incremental running test on a motorized treadmill (Run Race, Technogym, Gambettola, Italy) at an inclination of 1%. All participants were accustomed to treadmill running as it was extensively used during the pre-marathon training period. After 10 min warm-up at 70% of age-predicted maximal heart rate, the work protocol began at 9 km·h^-1 ^and the speed was increased by 1 km·h^-1 ^every minute so that exhaustion was reached in 8-12 min. Maximal oxygen uptake was considered to be the highest oxygen volume recorded during the last minute of exercise.

Achievement of VO_2max _was considered as the attainment of at least two of the following criteria:

1. a plateau in VO_2 _despite increasing speeds;

2. a respiratory exchange ratio above 1.10;

3. a heart rate (HR) ± 10 beats·min^-1 ^of age-predicted maximal HR (220--age).

Expired gases were analysed using a breath-by breath automated gas analysis system (VMAX29, Sensor medics, Yorba Linda, CA). The flow, volume, and gas analysers were calibrated before each test according to the manufacturer's instructions. Heart rates were measured during the incremental test using recordable Polar Vantage NV heart rate monitors (Polar Electro Oy, Kempele, Finland).

Individual maximal heart rates were taken as the highest heart rate recorded during the treadmill test.

Resting heart rate (HR_rest_) was measured after awakening with subjects in rested state (i.e. quiet room, supine position). The HR_rest _was assumed as the lowest 5 s value out of a 5 min monitoring. During marathon HR were assessed in each subject (Polar Vantage NV heart rate monitors, Polar Electro Oy, Kempele, Finland) and data were downloaded on a portable PC (Acer Aspire 5000, China) and analysed using the specific software (Polar ProTrainer 5, Polar Electro Oy, Kempele, Finland) and an electronic spread-sheet (Excel, Microsoft Corporation, U.S.). To quantify the internal physical load during marathon, we used the method of Banister et al. (1986) [52] for the calculation of the TRIMP. This method multiplies the duration of a training session by the average HR achieved during that session (percentage of heart rate reserve). The heart rate reserve is weighted by a multiplying factor (y), in a manner that reflects the intensity of effort. This y factor is based upon the exponential rise of blood lactate levels with the fractional elevation of exercise above HR_rest_. Thus, as exercise intensity increases, as indicated by the HR response, the weighting factor increases exponentially.

Participants were asked to refrain from all exercise and the use of alcohol, tobacco, and caffeine in the 48 h before testing. Subjects consumed their last meal at least three hours before treadmill testing and a record of the nutrient content was taken in order to provide the sufficient carbohydrate intake during the week before testing.

### Blood sampling

Blood samples were drawn the day before marathon and two hours after marathon from male recreational long-distance runners. Peripheral blood mononuclear cells (PBMCs) were isolated from whole blood samples by Ficoll-Hypaque gradient. Briefly, each 20-mL sample of anticoagulated whole blood was diluted 1:3 in PBS and layered onto Histopaque-1077. Following centrifugation at 1500 *g *for 20 minutes, the PBMC-containing interface was transferred to a 15-mL conical centrifuge tube and washed once in ice-cold PBS. The viability of the cells before and after marathon was measured using classic trypan blue dye exclusion. The pellets were used to extract DNAs and RNAs.

### DNA fragmentation assay

Cells were washed twice with phosphate-buffered saline (PBS) and lysed by addition of a hypotonic solution (1% NP-40 in 20 mM EDTA, 50 mM Tris-HCl pH 7.5). After centrifugation at 1600 ×g for 5 min, the supernatant was collected and the extraction was repeated with the same lysis buffer. The supernatants was brought to 1% SDS and treated with RNase A (final concentration 5 mg/ml) for 2 h at 56°C followed by digestion with proteinase K (final concentration 2.5 mg/ml) at 45°C for at least 6 h. Before hydrolysis, a further cleaning of DNA was performed by phenol-chloroform extraction, followed by three successive ethanol precipitations in 2 M ammonium acetate. Pellets were dried for 30 min and resuspended in 200 µl Tris-EDTA pH 8.0. Aliquots of 20 µl containing 10 µg DNA were electrophoresed in 1.5% agarose gel [53].

Subsequent 3' end-labeling of DNA, gel electrophoresis, and quantitation of DNA fragmentation were performed. Briefly, 500 ng of DNA prepared from samples were end-labeled with [α^32^P]-ddATP (Amersham) and terminal transferase (Boehringer-Mannheim) for 60 minutes at 37°C. Labeled DNA was loaded onto a 2% agarose gel, separated by electrophoresis and visualized by autoradiography.

### RNA isolation and Northern blot

Total RNA was isolated from samples using Trizol reagent (GIBCO) according to the manufacturer's instructions, and separated on 1% (w/v) agarose gel containing 1 × MOPS buffer [20 mM 3-(N-morpholino) propanesulfonic acid, 8 mM sodium acetate and 1 mM EDTA] and 2.2 M formaldehyde. Total RNA was blotted onto nylon membranes (Hybond N, Amersham, Braunschweig, Germany) and hybridized with ^32^P-different cDNA in a hybridization solution containing 50% formamide at 42°C overnight as previously described [54,55]. The excess ^32^P-probe was removed by stringent washing three times with 0.1× SSC and 1% SDS at 65°C for 30 min each. Hybridization signals were detected with a PhosphorImager (Biorad). The relative amount of mRNA level was quantified using a Gel-Doc phosphorimager and Quantity One software (Bio-Rad) and normalized by the intensity of β-actin.

### Statistical analysis

The results are expressed as means ± standard deviations (SD) and 95% confidence intervals (95% CI). Before using parametric tests, the assumption of normality was verified using the Shapiro-Wilk W-test. Pearson's product moment correlation coefficients were used on all subjects to examine correlations between variables. Student's paired t-test was used to determine any significant differences in physiological variables before and after marathon. The effect size (ES) was calculated to assess meaningfulness of differences. Effect sizes of above 0.8, between 0.8 and 0.5, between 0.5 and 0.2 and lower than 0.2 were considered as large, moderate, small, and trivial respectively [56]. Significance was set at 0.05 (p ≤ 0.05). A Bonferroni correction for the number of paired t-test was used. The resulting p-level was p ≥ 0.005. SPSS statistical software package (SPSS Inc., Version 13.0.1 for Windows Chicago, IL, USA) was used for all statistical calculations.

## Authors' contributions

GM carried out the design of the study, drafted and edited the manuscript. GM, MT, MAR reviewed and edited the manuscript. GM, MT, BP, MI, CD carried out Northern Blot. VM, AA PSS participated in the exercise study. VM performed the statistical analysis, and data interpretation. GM and MT conceived of the study and the manuscript. All authors read and approved the final manuscript.

## Supplementary Material

Additional file 1 **The anti and pro-apoptotic and SIRTs mRNAs in healthy amateur runners who did not participate in the marathon**. The results show the DNA fragmentation and the bax, bcl-2 SIRT1, SIRT3 RNA levels in six healthy amateur runners (who did not participate in the marathon) samples before and after marathon. Click here for file

Additional file 2 **Figure 1**. DNA laddering Click here for file

Additional file 3 **Figure 2**. Bax, bcl-2, SIRT1 and SIRT3 RNA levels were estimated by Northern Blot Click here for file
